# Suppression of GNAI2 message in ovarian cancer

**DOI:** 10.1186/1757-2215-7-6

**Published:** 2014-01-14

**Authors:** John R Raymond, Kathryn M Appleton, Jennifer Y Pierce, Yuri K Peterson

**Affiliations:** 1 Department of Drug Discovery and Biomedical Sciences, College of Pharmacy Medical University of South Carolina, 280 Calhoun St, QF415, Charleston, SC 29425, USA; 2 Department of Obstetrics and Gynecology, Medical University of South Carolina, Charleston, SC 29425, USA

**Keywords:** G-protein, Estrogen, cAMP, mRNA, GPCR, GNAI2, CREB, PCR, Ovarian cancer

## Abstract

**Background:**

Understanding the integration of hormone signaling and how it impacts oncogenesis is critical for improved cancer treatments. Here we elucidate GNAI2 message alterations in ovarian cancer (OvCa). GNAI2 is a heterotrimeric G protein which couples cell surface hormone receptors to intracellular enzymes, and is best characterized for its direct role in regulating cAMP response element-binding protein (CREB) function by decreasing intracellular cAMP through inhibiting adenylyl cyclase.

**Methods:**

We probed the Origene human OvCa array for the presence of polymorphisms and gene expression alterations of GNAI2 using directing sequencing and qPCR. These data were supported by database mining of the [NCBI NIH GSE:6008, GSE:14764, GSE:29450, GDS:4066, GDS:3297, GSE:32474, and GSE:2003] datasets.

**Results:**

No significant polymorphisms were found, including an absence of the *gip*2 oncogene. However, 85.9% of (506 of 589) OvCa patients had decreased GNAI2 message. Further characterization demonstrated that the GNAI2 message was on average decreased 54% and maximally decreased by 2.8 fold in clear cell carcinoma. GNAI2 message decreased in early stage cancer while message was increased compared to normal in advanced cancers. The changes in GNAI2 also correlated to deregulation of CREB, Fos, Myc, cyclins, Arf, the transition from estrogen dependence to independence, and metastatic potential.

**Conclusion:**

These data strongly implicate GNAI2 as a critical regulator of oncogenesis and an upstream driver of cancer progression in OvCa.

## Background

Elucidation of the conserved molecular pathologies leading to ovarian cancer (OvCa) initiation and progression are of great interest for targeted therapies. Most OvCa patients present with advanced and metastatic forms and little is known about the early pathophysiology leading to this widespread disease [1]. In the ovary there are multiple specialized cellular and histologic types which are often grouped together for simplicity, but represent several distinct cancers which have both conserved and unique susceptibilities to oncogenesis and therapeutics.

The majority of ovarian cancers are epithelial in origin, including serous, endometrial, mucinous, and clear cell carcinomas [2,3]. Papillary serous tumors are the most common and thought to be mediated through p53 mutations and loss of BRCA with possible origination in the fallopian tube. Endometrioid carcinomas are pleiotropic and can be either estrogen receptor (ER) positive or negative, and display variable alterations in p53, PTEN, Ras, and E-cadherin [4]. Clear cell ovarian cancer represents ~5% of cases. Clear cell tumors often have normal p53 but decreased ER and CD44 and present more frequently in patients with a personal or family history of endometriosis [3]. Mucinous tumors make up about 10% of cases and also frequently show p53 mutations, but are most distinct by acquiring frequent KRAS alterations and secreting estrogen [5]. The diversity of specific types of cancer and potential mechanisms indicates a critical need to identify conserved upstream regulators that also function as integrators of multiple signaling inputs.

In recent years, G protein coupled receptors (GPCRs) signaling cascades have come to light as primary mediators of oncogenic signaling by playing critical roles in inflammation, transformation, invasion, and metastasis [6,7]. Overactive signaling at the level of hormones, receptors, or G protein can initiate and potentiate cancer [8-11]. One of the principal G proteins, GNAI2 (Gα_i_2 protein), has pleotropic effects in regulating cellular viability and migration. A large number of vital hormones including epinephrine, dopamine, acetylcholine, somatostatin, angiotensin, and sphingosine-1-phosphate signal through the Gα_i_ pathway [12]. Gα_i_ is best described as being the inhibitory isoform of Gα that suppresses adenylate cyclase activity leading to decreased cAMP accumulation [13-15]. However, Gα_i_ is also known to regulate many other effectors including Src, ERK1/2, phospholipase-C, and monomeric GTPase’s like Rap [10,16-22]. For example, LPA stimulation of Gα_i_2 leads to activation of Src and Rac which is critical for invasive migration of ovarian cancer cells [23]. Indicative of a conserved mechanism, Gα_i_2 is also critical for migration in prostate, macrophage, and neutrophil cells [10,24].

OvCa specific alterations in GNAI2 have been detected using serial analysis of gene expression (SAGE) [8,25,26] and there is evidence that a portion of the patient population contains a R^179^C mutation in GNAI2 known as the *gip2* oncogene [13,24,27-29]. The R^179^C mutations cause the Gα_i_2 enzyme to be GTPase deficient, preventing signal termination, and causing Gα_i_2 to be constantly active. Decreasing the expression or inhibiting the activation status of the *gip2* oncogene has anti-cancer effects in cell culture models [24,27]. The *gip*2 oncogene was first described in OvCa, where it was present in 3 of 10 non-epithelial endocrine tumors of the ovary [28]. Further reports searching for *gip2* showed no *gip*2 in samples of 62, 18, 14, and 13 OvCa patients [29-32]. More recent *gip*2 searches in other cancers have also come up negative [27,33,34]. All of these data indicate GNAI2 could be a central mediator in altering cellular responses during cancer initiation and development [8]. We therefore conducted studies probing human patient mRNA samples to determine the specific alterations of GNAI2 in OvCa.

## Methods

### Origene human ovarian cDNA panels sequencing and real-time PCR procedure

TissueScan™ Disease Tissue qPCR Human Ovarian Arrays (OCAs) I-VI were obtained (OriGene Technologies, Rockville MD) for GNAI2 *gip*2 mutations detection (Arg^179^ replaced with either Cys or His) and differential message expression relative to normal tissue GNAI2 levels. The panels include carefully annotated but de-identified human patient samples at various stages of OvCa development. Each panel comes in duplicate: one panel for β-actin control (primers supplied) and the second for our gene of interest. Our GNAI2 primers were designed to complement the β-actin primer efficiency through optimization utilizing an OvCa cell line (SKOV3) to the recommended PCR parameters for the Origene ovarian cDNA real-time PCR plates.

GNAI2 mRNA relative quantification of ovarian tissue samples by real-time PCR was performed using the compatible Stratagene Mx4000 Real-time PCR System thermocycler (Agilent Technologies, La Jolla, CA). OrigeneTissueScan Disease Tissue qPCR Arrays (Origene Technologies, Inc., Rockville, MD) provide the normal and tumor ovarian cDNA samples. Reactions were prepared according to manufacturer’s instructions utilizing Maxima SYBR Green qPCR Master Mix (Fermentas, Glen Burnie, MD) employing cDNA specific primer sets as follows:

GNAI2: (forward) 5’-GCCTACTACCTGAACGACCT-3’.

(reverse) 5’-ATGATGGACGTGTCTGTGAACC-3’.

β-Actin: (forward) 5’-CAGCCATGTACGTTGCTATCCAGG-3’.

(reverse) 5’-AGGTCCAGACGCAGGATGGCATG-3’.

Real-time PCR for GNAI2 and β -actin parameters:

1 cycle → 50°C 2 min (Activation).

1 cycle → 95°C 5 min (Pre-soak).

40 cycles → 95°C 15 sec, 60°C 1 min (Amplification).

1 cycle → 95°C 1 min, 55°C 30 s, 95°C 30 s (Dissociation).

Dissociation curve analysis followed each real-time PCR procedure for confirmation of a single transcript amplification, and products were visualized by 1% agarose ethidium bromide gel electrophoresis to verify correct amplicon size. Relative quantization values were calculated utilizing the comparative threshold cycle method [35] with normalization to β-actin and determined relative to the normalized average non-cancerous tissue samples.

Gel purification was executed using 5 Prime Agarose GelExact Mini Kit (Promega, Madison, WI) according to manufacturer’s instructions. Purified GNAI2 products were submitted for sequencing utilizing our GNAI2 forward primer through Genewiz, Inc. (South Plainfield, NJ). Prior to graphical representation, data was normalized to gene-centric values, whereby the average global expression value between normal and cancer (all data points) was calibrated as zero. This was accomplished by using the equation $\left(\frac{\text{expression}\;\text{value}}{\text{global}\;\text{average}}-1\right)$.

### Human transcriptome meta-analysis

Datasets were acquired from The Cancer Genome Atlas (TCGA) using normal ovarian and ovarian cancer dataset values downloaded from cbioportal TCGA, Nature 2011, and GEO datasets [GSE:6008] [36], [GSE:14764] [37], [GSE:29450] [38], [GDS:4066] [39], and [GDS:3297] [40] from the NCBI. In GSE:6008, Hendrix et al. determined the significance of fibroblast oncogenesis driven by Wnt in ovarian tumors using gene expression microarrays [36]. In GSE:14764, Denkert et al. developed a 300 gene expression based ovarian cancer prognostic index [37]. In GSE:29450, Stany et al. used laser captured microdissection samples and expression microarrays to analyze clear cell histotype OvCa [38]. In GDS:4066 Spillman et al. investigated changes in gene expression upon OvCa treatment with estrogen using a mouse xenograft model [39]. In GDS:3297 Partheen et al. analyzed 54 stage III serous ovarian adenocarcinoma tumor samples using mRNA expression oligonucleotide microarrays [40]. None of these studies explicitly investigated GNAI2.

### Statistical analysis

Statistics were calculated using nonparametric statistical tests due to the greater accuracy of such tests in circumstances where Gaussian normality cannot be assumed, and with only a ~5% error when used on Gaussian data [41]. Kruskal-Wallis and Mann-Whitney rank-sum tests were applied to all expression data unless otherwise noted. In one instance, GSE:6008 staging data was tested using an ANOVA under Gaussian assumptions due to the data passing Anderson-Darling normality tests. Gaussian statistics were used for histology data due to each staging group’s indication of normality according to the Anderson-Darling test. All data were analyzed using GraphPad Prism and Microsoft Excel. When appropriate, data was normalized to gene-centric values, whereby the average global expression value between normal and cancer (all data points) was calibrated as zero.

### Ethics approval

These studies were designated Not Human Research by the Medical University of South Carolina Institutional Review Board (Pro 24780) according to the Code of Federal Regulations (45CFR46) due to anonymized handling and retrospective analysis of data.

## Results

### Origene human ovarian cDNA panels sequencing

We began by investigating the human Origene ovarian cancer array (OCA) using direct sequencing within the coding region of GNAI2 transcripts. We found no mutations within 192 samples. Analysis of the Cbioportal database indicated one missense mutation in 489 samples (A^114^T). The 1000genomes database has a single silent polymorphism in 1000 samples [42]. These all differ from the known activating mutations of GNAI2: R^179^C and Q^205^L [13].

### Origene human ovarian cDNA panels real-time PCR

The low prevalence of *gip2* is surprising as the *gip2* mutation is well characterized as transformative. This leaves the possibility that there were changes in gene expression. We probed the OCA using qPCR for GNAI2. The OCA demonstrated high variability in GNAI2 expression, but with the surprising result that the majority of cancer patients underexpress GNAI2 (Figure 1A/C). The mean for normal ovarian tissue was 0.42 ± 0.11 while the mean in OvCa was -0.07 ± 0.04 (p < 0.004). These qualitative data revealed 141 individuals, or 85.5% of cancers, underexpressed GNAI2 compared to the normal within the Origene OCA. Seventy two samples (43.6%) underexpressed below the -0.28 absolute minimum expression threshold of normal patients.

**Figure 1:** **GNAI2 message is suppressed in ovarian cancer. A**. Rank order of GNAI2 expression of Origene OCA. Normal n = 27, Cancer n = 165. **B**. GNAI2 expression from NIH NCBI TCGA, Nature 2011. Normal n = 8, Cancer n = 315. **C**. Scatter plot of **A**. * = cancer specific underexpression in 58% of patients. p < 0.004. **D**. Scatter plot of **B**. * = Nonparametric p < 0.003 Normal n = 8, Cancer n = 315. E. and **F**. GNAI2 expression of NCI60 samples. **E**. Data derived from GSE32374. **F**. Data derived from GSE2003. Expression presented as normalized gene centric values derived from ∆∆CT with variance presented as 95% CI.

### Human GNAI2 transcriptome meta-analysis

To further confirm our results, we analyzed data from the NIH GEO database. The Nature 2011 dataset confirms the trend and indicated 266 samples, or 84.4% of cancer, were below the normal mean expression value of 0.38 ± 0.09 (p < 0.004) and 84 samples, or 26.7%, were below the absolute minimum expression value of -0.21 from disease free patients (Figure 1B/D) [43]. All 10 cancer samples (100%) were found to underexpress with regard to normal in GSE:29450, and 89 samples (89.9%) were below normal GNAI2 message expression in GSE:6008. The general trend in the magnitude of expression profiles was reflected in the variance in expression from three of the NCI60 cell lines. In this data set we found six OvCa cell lines with a mean difference in GNAI2 expression of about one fold (Figure 1E/F). OVCAR4 cells have the lowest GNAI2 expression (-0.39 fold) while OVCAR8 had the highest (+0.23) and SKOV3 cells were intermediate (-0.09).

GNAI2 expression was significantly reduced in cancer patients (n = 505 reduced/589 total); however, the variability in human expression, cellular origin, or cancer progression from other cancer arrays was of interest. We analyzed cell type and staging data for GNAI2 in OvCa patients utilizing diverse publicly available gene transcription datasets with available GNAI2 expression levels.

### Histology and staging analysis

In the GSE:6008 and GSE:14764 datasets, GNAI2 expression was decreased in all types of OvCa but was distinct among histological types of OvCa (Figure 2A/B). Clear cell and mucinous cancers had the greatest reduction in message amongst cancer cell types, with a mean of 2.91 ± 0.05 (p < 0.005) for clear cell and 2.92 ± 0.07 (p < 0.03) for mucinous for a change of 0.37 fold versus 3.28 ± 0.05 (p < 0.01) for normal tissue samples. Endometrioid and serous carcinomas were also depressed and significantly below normal samples. Dataset GSE:29450 confirmed the trend of underexpression of GNAI2 in ovarian cancer cells. In particular, all clear cell cancer samples expressed below the mean expression in non-cancerous tissue (p < 0.0001) (Figure 2C).

**Figure 2:** **GNAI2 expression correlates with ovarian cancer tissue type. A**. Data derived from GSE6008 normal n = 4, mucinous n = 13, clear cell n = 8, endometrioid n = 37, serous n = 41. Nonparametric normal and clear p < 0.005, normal and mucinous p < 0.03, normal and endometrioid p < 0.02, normal and serous p < 0.05. Expression is presented as *HPRT1* normalized ∆∆CT. **B**. Data derived from GSE14764. Clear cell n = 2, endometrial ovarian n = 7, serous n = 68. Kruskal-Wallis ANOVA p < 0.005. Expression is presented as Affymetrix MAS 5.0 signal intensity **C**. Data derived from GSE29450. Normal n = 10. Clear Cell n = 10. Nonparametric p < 0.0001. Values reported as RMA signal intensity. **D**. GNAI2 expression correlates with estrogen sensitivity. Data derived from GDS4066, ER + n = 7, ER- n = 8. Nonparametric p < 0.006. Values reported as RMA signal intensity.

The relationship between GNAI2 and endocrine control was also of interest. We therefore analyzed GNAI2 expression according to estrogen receptor status. GNAI2 expression varies significantly between ER + versus ER- cells in dataset GDS:4066 (Figure 2D). ER + cells expressed 7.73 ± 0.12 GNAI2 whereas ER- cells expressed 8.24 ± 0.08 (p < 0.006 between ER + and ER-) for a decrease of 0.51 fold.

GNAI2 expression also correlates with tumor stage independent of cell histology (Figure 3). In GDS:3297 dataset stage IIIB GNAI2 expression was -0.40 ± 0.20 and significantly lower than IIIC expression of -0.11 ± 0.12 (p < 0.04, Figure 3A). These results were paralleled in the TCGA Nature 2011 dataset where IIIA OvCa had the lowest mean expression of -0.47 ± 0.22 (p < 0.009) while late stage cancer, IIIC and IV, had means of 0.02 ± 0.02 and -0.02 ± 0.06, respectively (Figure 3B). In the GSE:6008 dataset, which uses a different scale than stage IIC OvCa had the lowest expression of 9.38 ± 0.27 and stages III, IIIC, and IV were statistically distinguishable via (p < 0.03 via Kruskal-Wallis ANOVA) (Figure 3C).

**Figure 3:** **GNAI2 expression correlates with tumor stage. A**. Data derived from GDS3297. IIIB n = 9, IIIC n = 23. Nonparametric p < 0.04 **B**. Data derived from TCGA, Nature 2011. Normal n = 8, IIA n = 2, IIB n = 4, IIC n = 8, IIIA n = 4, IIIB n = 14, IIIC n = 230, IV n = 53. Kruskal-Wallis p < 0.02. Normal versus IIIA nonparametric p < 0.009, IIIB Nonparametric p < 0.006, IIIC Nonparametric p < 0.004, IV Nonparametric p < 0.007. **C**. Data derived from GSE6008: stage III n = 2, IIIC n = 25, IV n = 5. Kruskal-Wallis ANOVA p < 0.03, Gaussian ANOVA p < 0.05, Gaussian III vs. IV p < 0.04, Gaussian IIIC vs. IV p < 0.05. Anderson-Darling Normality for IIIC p > 0.6 and for IV p > 0.9. Stage IIIC and stage IV were also statistically different using a parametric T-test. Expression is presented as *HPRT1* normalized ∆∆CT. **D**. Methylation of GNAI2 gene correlates inversely with GNAI2 message expression. Methylation values reported as beta values.

The presence of increased gene methylation and decreased message would suggest regulated gene silencing. We therefore wanted to determine if methylation was a possible mechanism for the alterations in GNAI2, as opposed to upstream regulation of message. The Nature 2011 HM27 data revealed a correlation between GNAI2 gene methylation and cancer staging although the means were not statistically significant (Figure 3D). Methylation increased with cancer stage and was especially pronounced in several patients with class IIIC tumors. These data are congruent with the GNAI2 promoter being regulated through transcriptional gene control.

### Transcriptome meta-analysis downstream of GNAI2

The consequence of downregulating GNAI2 leads to disregulation of adenylyl cyclase, hyperaccumulation of cAMP, thereby causing hyperactivation of CREB. Activation of CREB then alters gene transcription of cAMP response elements (CRE) leading to altered expression of CRE responsive genes including other transcription factors like Fos and Myc as well as other oncogenes like cyclins and Arf [44-46]. We therefore analyzed the available datasets for alterations in CREB, and CRE responsive genes. Dataset GSE6008 indicated CREBL2, Fos, and Myc were underexpressed (Figure 4). CREBL2 showed lowest expression in endometrioid ovarian cancer, and was found to express below the normal mean of 3.66 ± 0.03 for the following OvCa histotypes: clear cell at 3.25 ± 0.04 (p < 0.005), mucinous at 3.29 ± 0.03 (p < 0.004), endometrioid at 3.22 ± 0.03 (p < 0.003), and serous at 3.24 ± 0.02 mean expression (p < 0.002) (Figure 4A). Fos expressed below the normal mean value of 4.31 ± 0.02 in all histotypes as follows, with minimal expression demonstrated in clear cell: clear cell at 3.38 ± 0.20 (p < 0.005), mucinous at 3.71 ± 0.14 (p < 0.04), endometrioid at 3.43 ± 0.08 (p < 0.002), and serous at 3.56 ± 0.06 (p < 0.002) (Figure 4B). Myc expression in ovarian cancers was lower than normal, with the mean expression of 2.82 ± 0.13 (p < 0.005) for clear, 3.35 ± 0.14 (p < 0.04) for mucinous, 3.38 ± 0.06 (p < 0.02) for endometrioid, 3.47 ± 0.06 (p < 0.07) for serous, and 3.78 ± 0.04 for normal tissue (Figure 4C). This underexpression is indicative of feedback gene repression due to hyperactivation of the signaling pathway.

**Figure 4:** **CRE effects in ovarian cancer.** Data derived from GSE6008. Normal n = 4, mucinous n = 13, clear cell n = 8, endometrioid n = 37, serous n = 41. **A**. Nonparametric normal and clear p < 0.005, normal and mucinous p < 0.004, normal and endometrioid p < 0.003, normal and serous p < 0.002. **B**. Nonparametric normal versus endometrioid p < 0.03, normal and serous p < 0.004 **C**. Nonparametric normal and clear p < 0.005, normal and mucinous p < 0.004, normal and endometrioid p < 0.002, normal and serous p < 0.003. **D**. Nonparametric normal and endometroioid p < 0.027, normal and serous p < 0.004 **E**. Nonparametric normal and clear p < 0.005, normal and mucinous p < 0.004, normal and endometrioid p < 0.002, normal and serous p < 0.003. **F**. Nonparametric normal and clear p = 0.004. **G**. Nonparametric normal and clear p < 0.05, normal and mucinous p < 0.02, normal and endometrioid p < 0.008, normal and serous p < 0.002. **H**. Data derived from from NIH NCBI TCGA, Nature 2011. Normal n = 8, stage IIA n = 3, IIB n = 4, IIC n = 16, stage IIIA n = 7, stage IIIB n = 21, stage IIIC n = 353, stage IV n = 79. Nonparametric normal and stage IIA p < 0.01, normal and stage IIB p < 0.005, normal and stage IIC p < 0.001, normal and stage IIIA was p < 0.03, normal and stage IIIB p < 0.002, normal and stage IIIC p < 0.0001, normal and stage IV p < 0.0001. **I**. Data derived from NIH NCBI TCGA, Nature 2011. Stage IIB n = 4, IIC n = 8, stage IIIA n = 4, stage IIIB n = 14, stage IIIC n = 230, stage IV n = 53.

We found Cyclin A1, Cyclin D1 and Arf4L, which are all downstream of GNAI2/cAMP/CREB, were overexpressed. Cyclin A1 was significantly overexpressed in both endometroioid, with a mean of 2.95 ± 0.09 (p < 0.027), and serous 3.19 ± 0.07 (p < 0.004) compared to normal 2.31 ± 0.07 in dataset GSE:6008 (Figure 4D). Cyclin D1 was overexpressed in comparison to normal in all histotypes (Figure 4E). Normal expression was 2.37 ± 0.07, compared to clear 2.89 ± 0.07 (p < 0.005), mucinous 3.26 ± 0.09 (p < 0.004), endometrioid 3.27 ± 0.06 (p < 0.002), and serous 3.10 ± 0.07 (p < 0.003). Arf4L overexpressed in clear cell, with a mean of 3.37 ± 0.03 versus normal’s 3.04 ± 0.04 (p = 0.004), and was not significantly different from normal in mucinous, endometrial or serous OvCa (Figure 4F). Both the histology and staging data from GSE:6008 and Nature 2011, respectively, showed that MAPK10 was decreased in expression compared to normal which was consistent as its established role is as a tumor suppressor [47]. MAPK10 had lowest expression in serous cancer. Expression in clear cell was 2.96 ± 0.03 (p < 0.05), in mucinous 2.95 ± 0.04 (p < 0.02), in endometrioid 2.919 ± 0.02 (p < 0.008), and in serous 2.84 ± 0.02 (p < 0.002). All of these were below the normal expression of 3.12 ± 0.06 (Figure 4G). The Nature 2011 dataset yielded staging data correlations with MAPK10 expression where all stages of cancer underexpressed MAPK10 versus normal’s mean of 1.08 ± (Figure 4H). Stage IIA expression was 0.15 ± 0.12 (p < 0.01), stage IIB was -0.17 ± 0.18 (p < 0.005), stage IIC -0.15 ± 0.12 (p < 0.001), stage IIIA was 0.25 ± 0.40 (p < 0.03), stage IIIB was 0.05 ± 0.14 (p < 0.002), stage IIIC was -0.03 ± 0.03 (p < 0.0001), and stage IV -0.17 ± 0.05 (p < 0.0001). In the Nature 2011 dataset, Fos expression did not significantly vary with staging (Figure 4I).

## Discussion

We interrogated human OvCa for the presence of polymorphisms and altered gene expression of GNAI2. GNAI2 functions as a critical upstream regulator of OvCa through suppression of cAMP, CREB activity, CRE function, and gene regulation. The increase in cAMP is necessary for rapid growth and activation of CREB, promoting angiogenesis, and protecting cancer cells from apoptosis [48]. The *gip2* activating polymorphisms in GNAI2 were not present in 681 patient samples (n = 192 for Origene and n = 489 from Nature 2011), reaffirming previous data that the *gip*2 oncogene is rare in the human population. However, when we aggregate our OvCa data with published array data in datasets GSE:6008, Nature 2011, and GSE:29450, a consistent 86% of OvCa patients had decreased GNAI2 message levels with respect to normal. Further characterization indicated a maximal decrease of GNAI2 expression in clear cell phenotype. The Nature HM27 arrays confirm methylation of the GNAI2 gene, and Cbioportal data discounts the possibility of gene deletion yielding false positives for methylation. Methylation of GNAI2, which suppresses gene transcription, generally increased with cancer stage and hypermethylation was observed in 34.6% of patients with Stage IIIC tumors (n = 353, mean = 0.09 ± 0.01).

GNAI2 message correlated with cancer stage and mean message levels returned to normal (or overexpressed) levels in most advanced cancer stages. These data indicate GNAI2 alterations correlate with histologic type and cancer stage. In late stage cancer, cells could switch signaling such that Gα_i_ is uncoupled from the regulation of cAMP/CREB dependent proliferation to CREB independent/migratory phenotypes [49,50]. G protein regulatory (GPR)/Goloco motif-containing proteins, which uncouple Gα_i_ from GPCRs and prevent GDP release have also been implicated in the regulation of cell division and differentiation [51-54].

GNAI2 message decreased on average 54% (0.5 fold) from normal. The likely reason GNAI2 was not picked up in many transcriptome studies was that most searches emphasize genes with large changes in pathological expression (<200% or two fold). However, genes of high importance can cause dramatic effects through small expression variations, especially in G protein mediated amplification cascades. As the body of data grows, more studies are also finding a link between cancer and aberrant GPCR/ER expression and/or activation [11,55,56]. GNAI2 has the unique ability to link GPCR and estrogen signaling through its ability to suppress cAMP [57]. A decrease in Gα_i_ in cancer should increase the efficacy of estrogen and GPCR mediated increases in cAMP production. This may be of particular importance in cancers thought to have an origin in estrogen mediated processes such as the link between clear cell carcinoma and endometriosis. Regardless of the pathway, higher cAMP in cancer corresponds to poorer prognosis [58]. Recent discoveries regarding proteins such as NOTCH, Fos, and E-cadherin also indicate that there is a subset of critical proteins that can function as either oncogenes or tumor suppressors, depending on cell type and/or tumor progression [59]. The decrease in GNAI2 in cancer patients suggests that its functional role in humans is pleiotropic and that GNAI2 can also function as a tumor suppressor depending on the cellular context.

## Conclusions

GNAI2 was found to be underexpressed in the majority of the ovarian cancer patient population. By being situated upstream of regulatory mechanisms that control both proliferation and migration, GNAI2 could prove to be a useful diagnostic indicator or potential therapeutic target in ovarian cancer. However, our analyses did not follow the clinical outcomes of the disease and therefore more research must be done to determine if GNAI2 has prognostic value. These data provide a strong rationale for GNAI2 being a central player in ovarian epithelial cell fate decisions during oncogenesis.

## Abbreviations

CRE: CAMP response elements; CREB: CAMP response element-binding protein; ER: Estrogen receptor; GPCR: G-protein coupled receptor; GPR: G-protein regulatory; OCA: Ovarian cancer array; OvCa: Ovarian cancer; PCR: Polymerase chain reaction; SAGE: Serial analysis of gene expression; TCGA: The Cancer Genome Atlas.

## Competing interest

The authors declare that they have no competing interests.

## Authors’ contributions

YKP managed the overall project. All authors participated in research design and contributed to the writing of the manuscript. KMA designed and performed the PCR analysis. JRR performed the database meta-analysis. All authors read and approved the final manuscript.
